# Does Fine Color Discrimination Learning in Free-Flying Honeybees Change Mushroom-Body Calyx Neuroarchitecture?

**DOI:** 10.1371/journal.pone.0164386

**Published:** 2016-10-26

**Authors:** Frank M. J. Sommerlandt, Johannes Spaethe, Wolfgang Rössler, Adrian G. Dyer

**Affiliations:** 1 Department of Behavioral Physiology and Sociobiology, Biozentrum, University of Würzburg, Am Hubland, Würzburg, Germany; 2 School of Media and Communication, RMIT University, Melbourne, Victoria, Australia; Universitat Regensburg, GERMANY

## Abstract

Honeybees learn color information of rewarding flowers and recall these memories in future decisions. For fine color discrimination, bees require differential conditioning with a concurrent presentation of target and distractor stimuli to form a long-term memory. Here we investigated whether the long-term storage of color information shapes the neural network of microglomeruli in the mushroom body calyces and if this depends on the type of conditioning. Free-flying honeybees were individually trained to a pair of perceptually similar colors in either absolute conditioning towards one of the colors or in differential conditioning with both colors. Subsequently, bees of either conditioning groups were tested in non-rewarded discrimination tests with the two colors. Only bees trained with differential conditioning preferred the previously learned color, whereas bees of the absolute conditioning group, and a stimuli-naïve group, chose randomly among color stimuli. All bees were then kept individually for three days in the dark to allow for complete long-term memory formation. Whole-mount immunostaining was subsequently used to quantify variation of microglomeruli number and density in the mushroom-body lip and collar. We found no significant differences among groups in neuropil volumes and total microglomeruli numbers, but learning performance was negatively correlated with microglomeruli density in the absolute conditioning group. Based on these findings we aim to promote future research approaches combining behaviorally relevant color learning tests in honeybees under free-flight conditions with neuroimaging analysis; we also discuss possible limitations of this approach.

## Introduction

Bees are important pollinators of flowers and, in return, flowers often provide a vital source of nutrients for bees [1, 2]. Besides olfactory cues [3], bees use a variety of visual information [4, 5] to find rewarding flowers. However, in complex natural environments not all plants present flowers that are rewarding and some flowers mimic true rewarding flowers to incidentally receive flower visits by insects to facilitate pollination [6, 7]. This complex foraging situation places demands on the visual processing of bees for fine discriminations [8], but to date there is a relative dearth of information about how the sensory processing system of bees facilitates such rich visual capabilities as have been observed in psychophysical studies.

Color is one of the most important features used by honeybees to identify flowers as potential food sources [9–15]. To enable highly efficient foraging, bees not only have to perceive the color information, but also have to learn this information [16, 17] and retrieve it after days or even weeks [18]. Honeybees are able to learn colors within their perceptual range (from 300 nm to 650 nm), although with varying efficiencies depending upon wavelength ([11, 17] reviewed in [19]). However, the performance level when discriminating two colors is highly dependent on the way in which stimuli are encountered in a foraging situation [8]. Discrimination of perceptually similar colors requires differential conditioning with target and distractor stimuli. In contrast, when target colors are learnt in isolation with absolute conditioning only a coarse level of color discrimination develops, i.e. the discrimination of perceptually different colors can be achieved [14, 20]. This not only suggests different levels of behavioral plasticity in bee color learning, but also different underlying neuronal processes. A first step towards understanding these mechanisms is to identify the neuropils where such visual information may be processed and stored in a bee brain. Due to the complexity of visual computations, several brain regions might be involved, either in parallel or via serial processing of such information [4, 21–23].

Potentially essential neuropils are the paired mushroom bodies (MB) which have been identified as sensory integration centers that facilitate associative learning and (long-term) memory formation [24–30]. In honeybees, the MBs contain a high number of neurons (ca. 170,000–184,000 Kenyon cells per MB [31]; reviewed in [26, 32]) and take up a large part of the brain volume compared to other neuropils. Recent studies have shown that age, behavior and social environment may affect volumetric properties of the MB and its substructures [33–35]. The four cup-shaped calyces (one median and lateral calyx per MB and brain hemisphere) represent the sensory input regions of the MBs. These structures are sub-divided into three modality-specific compartments comprising (i) the lip, receiving olfactory information from the antennal lobes, (ii) the collar, receiving visual information from the optical lobes, and (iii) the basal ring, a region that integrates olfactory and visual information [21, 36–39]. Neuronal circuits within a calyx are organized in distinct microglomeruli (MG), synaptic complexes consisting of a single presynaptic bouton from the axon terminals of a projection neuron that is surrounded by numerous postsynaptic dendritic spines of MB intrinsic neurons, the Kenyon cells [29, 32, 40, 41]. Additionally, (GABAergic) MB feedback neurons and modulatory aminergic neurons project to the calyces and contribute to the microcircuits of the MG [34, 42]. The MG synaptic circuits are characterized by a high degree of structural plasticity, as changes in the distribution (or density) of the synaptic complexes are found to be associated with age [34, 35], light exposure [43], and the formation of olfactory long-term memory [28]. The late (stable) form of olfactory long-term memory lasts for 2 days up to lifetime and depends on protein synthesis [44, 45]. This was shown to be accompanied by an increase in MG densities and total numbers in the olfactory lip region of the MB calyx [28, 30].

It is unknown whether fine color discrimination and the formation of visual long-term memory is also processed in the MBs and, thus, might affect (or is affected by) the MB calyx neuronal network and synaptic structure. In bees, the visual collar region of the MB calyces is innervated by projection neurons deriving from inner medulla and inner lobula layers ([46], reviewed in [4]). Thus, major effects in visual memory formation should take place in the visually innervated collar, although little is known for color learning in free flying bees. Based on this assumption, we aimed to test the following two hypotheses: First, in analogy to findings in olfactory learning experiments [28], we propose that the formation of a new visual memory should be associated with an increase in MG density in the MB collar. Second, the strength of the effect on MG density should be correlated with the complexity of the visual learning task, i.e. compared to an easy absolute conditioning task, bees that learn to discriminate between a pair of perceptually similar colors in a differential conditioning paradigm have to learn more stimulus features, and thus more neuronal circuits may be involved. To investigate whether the MG synaptic network is shaped by visual learning and depends on the level of complexity of a learning task, honeybee foragers were individually trained in either absolute or differential conditioning with two perceptually similar colors and subsequently tested for color discrimination abilities in a choice test. MB characteristics (volume and MG number and density) were measured after three days (to allow long-term memory formation) and tested for potential correlation with behavioral performance. With this study we aim to provide a first step towards understanding potential neuronal mechanisms underlying color learning and memory formation in bees under natural free-flying conditions.

## Materials and Methods

### Behavioral Color Conditioning

Experiments were conducted with the European honeybee (*Apis mellifera carnica*) maintained in a colony located at the Campus Hubland Nord of the Julius Maximilian University (Würzburg, Germany). A feeding site (gravity feeder; e.g. as shown in [47]) was positioned 25 m away from the colony, from which foragers were allowed to collect 5–10% (w/w) sucrose solution *ad libitum*. Individual bees were transferred (by means of a Plexiglas^®^ spoon with a drop of sucrose solution) from the feeding site to a test site 6 m away, where they received 25% sucrose solution and were individually color marked on their thorax. Each bee was trained and tested individually, which lasted approx. 90–120 min per individual.

Color stimuli were made from cardboard (6 x 8 cm2; Tonpapier no. 32 [turquoise] and 37 [blue], Baehr, Germany; as used in [18, 48]) that appear to a human observer turquoise and blue, respectively. The stimuli were covered with matt lamination foil (ARGO SA, 80–393 Gdansk, Poland) and attached to freely rotating hangers with a landing platform, presented on a vertical, circular and rotatable plastic screen of 50 cm diameter (as described in [49]; in the following referred to as "rotating screen"). This set-up allowed an efficient rearrangement of the stimuli to avoid location learning, and hanger replacement to avoid olfactory markings [50]. The spectral reflectance of the stimuli was measured with a JAZ S1 spectrometer (Ocean Optics; Fig 1A) and color loci were calculated in a hexagon color space [51] (Fig 1B). The color distance (considering the grey background color of the rotating screen) between turquoise and blue was 0.075 hexagon units, which is sufficiently large to be discriminated by bees [52, 53]. Target stimuli (CS+) were reinforced by 10 μl of 25% sucrose solution (US+) placed on the landing platform, whereas distractor stimuli (CS-) contained 10 μl of pure water (US-).

**Fig 1:** Color stimuli qualities. **A** Spectral reflectance of stimuli. **B** Loci of color stimuli in a color hexagon. The cross marks the location of the blue stimulus, while the triangle indicates the location of the turquoise stimulus. The hexagon’s center is indicated by the dot. See text for details.

Individual bees were randomly assigned to one of three treatment groups: one group of bees received absolute conditioning with two rewarded target hangers (either blue or turquoise) and two unrewarded grey hangers being of the same grey as the background. We are aware, that due to the experimental setup, the bees in this group have to discriminate between two types of hangers (colored vs. background-like grey) and hence are confronted with an “easy” differential conditioning task. Nevertheless, in regard to the chromatic information provided by the stimuli, one can retain the terminology of absolute conditioning [54]. This is consistent with literature about absolute visual conditioning in free-flying bees, where some form of alternative is presented to allow quantification of choices [14]. A second group of bees was trained using differential conditioning, i.e. these bees had to discriminate between two blue and two turquoise hangers; on one color (either blue or turquoise) sucrose solution (CS+) was provided and the other (remaining) color (CS-) was presented with pure water. A third control group (grey group) was confronted with two grey hangers providing sugar solution and two grey hangers offering pure water, thus these bees could not use any (visual) cues to discriminate the rewarded from the unrewarded stimuli, and thus we expected no color learning effect at all.

Each of the 43 bees was trained for a total number of 50 decisions (fulfilled with approx. 15–20 foraging bouts). A decision was counted when a bee made any contact with the landing platform or solution. All groups and stimuli were tested in a pseudorandomized order. Sample size per experimental group is given in figure descriptions in the results part.

We are aware, that sensory exposure can affect microglomeruli distribution [35, 43]. However, with the recruitment procedure from a feeder dish we ensured that all tested bees were of the same ontogenetical state (foragers) with fully maturated brains [35]. Moreover, due to a random assignment of individual bees to the experimental groups, potential learning-dependent changes should not be masked by variation due to age.

### Choice Test

Following the training phase, each bee was allowed to imbibe sucrose solution on the next visited CS+ hanger until it was satiated and returned to the hive. After returning to the test site, each bee (of all three tested groups) was individually tested for its color preference in an unrewarded choice test, where two hangers with blue stimuli and two hangers with turquoise stimuli were presented on the rotating screen in a pseudorandom arrangement. The first 20 choices were counted, with a choice being scored when the bee touched or landed on a hanger.

### Bee maintenance following behavioral testing

To allow for complete long-term memory formation (which includes protein synthesis, [44]), all bees that completed the behavioral experiments were maintained for three days in constant darkness at 27°C and 60–70% humidity. An additional group of bees, termed as feeder control group, was caught directly from the gravity feeder, to obtain a control group with the same ontogenic state (forager bees), but without experience of the rotating screen setup (and its operant requirements), and was also put for three days into the dark. For this purpose, bees were caged individually in polystyrene tubes (6 cm in length and 2 cm diameter), closed by foam plugs and furnished with a 1 x 4 cm piece of wax panel and a feeding dish, containing a water-solved mixture of glucose and fructose. Due to the free-flying test conditions, bees were not behaviorally tested for long-term memory after three days.

### Immunohistochemistry

After maintaining the bees for three days, synaptic complexes in the mushroom body calyces were visualized by means of immunohistochemistry using whole-mount preparations as described by Groh *et al*. [34] and Muenz *et al*. [35]. Briefly, each bee was chilled on ice and the head capsule was opened frontally. After removal of tracheae and secretory glands, the heads were immediately transferred to 4% formaldehyde (FA) in phosphate-buffered saline (PBS), immersed overnight at 4°C and then washed in PBS (3 x 10 min). The heads were then fixed in dental wax and dissected in PBS. The isolated brains were first permeabilized in 2% Triton X-100 (Tx) in PBS for 10 min, then washed in 0.2% PBS-Tx (2 x 10 min) and eventually blocked in 2% normal goat serum (NGS) in 0.2% PBS-Tx for one hour at RT. For anti-synapsin immunohistochemistry, brains were incubated with the monoclonal primary antibody against the *Drosophila* synaptic vesicle associated protein synapsin I (SYNORF1; kindly provided by Dr. E. Buchner, University of Würzburg, Germany), diluted 1:50 in 0.2% PBS-Tx with 2% NGS for four days at 4°C. After rinsing in PBS (5 x 10 min), brains were incubated in CF488-conjugated goat anti-mouse secondary antibody (1:250) in PBS with 1% NGS for four days at 4°C. Brains were finally washed in PBS (5 x 10 min), dehydrated in an ascending ethanol series (30%, 50%, 70%, 90%, 95%, 3 x 100%, each step lasting 10 min) and cleared and mounted in methyl salicylate.

### Laser scanning confocal microscopy, processing and data acquisition

Whole mount preparations were examined using a laser scanning confocal microscope (Leica TCS SP2 AOBS, Leica Microsystems AG, Wetzlar, Germany) with optical sections being taken at a resolution of 1,024 x 1,024 pixels (Fig 2A). For calyx reconstruction and volume measurements, optical sections at 5 μm intervals (HC PL APO objective lens: 10x/0.4 NA imm; digital zoom 3.5–4.0) were taken entirely through one of the randomly chosen medial calyces, and for analysis of MG density, high resolution scans were taken from the lip and dense collar region in randomly chosen anterior-posterior direction up to a depth of 10 μm at 0.5 μm intervals (63x/1.4 NA imm, digital zoom 2; Fig 2B and 2C). Digital image stacks were further processed by means of 3D software (AMIRA 5.3; FEI Visualization Sciences Group, Düsseldorf, Germany). Calyces were digitally reconstructed for volumetric analysis by manually tracing the neuropil boundaries of the lip, collar (divided in dense and loose region; [34]), and basal ring on each optical section with subsequent interpolation (Fig 2D). The number of MG (estimated by counts of large synapsin-positive boutons) was analyzed in cubic volumes of 1,000 μm^3^ in three regions: two cubes each in the medial and lateral antennal lobe tract (m- and lALT; nomenclature after [55]) innervated lip region, and three cubes in the dense collar region (Fig 2B and 2C; see [34] for details). All counts were done in a blind manner without knowledge about the experimental group, and MG number was region-specific averaged per individual. To obtain estimation about the region-specific total MG number per calyx, mean MG number per 1,000 μm^3^ cube was multiplied by the subregion’s volume.

**Fig 2:** Synapsin immunostaining and 3D calyx reconstruction of a forager honeybee brain. **A** Confocal image of a frontal section through the brain after whole-mount immunolabeling for synapsin. Calyx volume and MG density were quantified in one of the medial calyces (mCA). In the magnified view of the lip (**B**) and the collar (**C**), synapsin-labeled projection neuron boutons (MG) were counted in defined volumes (1000 μm^3^; yellow cubes) in three regions: mALT innervated lip, lALT innervated lip, and dense collar (dCO). **D** Cross section of the volume reconstruction of the mCA rendered from confocal image stacks. AL, antennal lobe; BR, basal ring; mCA, medial calyx; lCA, lateral calyx; CX, central complex; dCO, dense collar; lCO, loose collar; LA, lamina; LO, lobula; MB, mushroom body; ME, medulla; PED, peduncle. Axes: ca, caudal; le, left; ri, right; ro, rostral. Scale bar in **A** is 500 μm, in **B** (and **C**) 25 μm, and in **D** 100 μm.

### Statistical analyses

For the behavioral experiments, the proportion of correct decisions (decision towards CS+) was calculated considering blocks of 10 trials for the three respective experimental groups, and compared to random choice level (0.5) by means of a Wilcoxon test after arcsin square root transformation. For the “grey” control group, two out of four grey stimuli were at the beginning of the experiment randomly defined as “target” and the remaining two as “distractor” (non-rewarded CS-) to record the proportion of virtually “correct” landings. Group performance in the color choice test was compared to random choice level on the basis of the foragers’ proportion of correct decisions using a Wilcoxon test after arcsin square root transformation. For the “grey” control group, the blue stimulus was declared as “correct” and the turquoise stimulus was declared as “incorrect”, to obtain the proportion of “correct” landings. This group additionally served as a test group for a potential preference towards either the blue or the turquoise stimuli. Volumes of brain regions and MG numbers were compared among experimental groups using Kruskal-Wallis-H test. Possible differences between MG number of lALT and mALT region in the MB lip was calculated using Mann-Whitney-U test. Correlation between learning performance (based on the individual’s number of correct landings during the 50 conditioning trials) and number of MG was calculated by means of Spearman correlation analysis.

## Results

### Color conditioning and choice test

Color learning (Fig 3) in the absolute conditioning group occurred rapidly, and bees were able to choose the target color to a significant extent already within the first block (trial 1-10: 0.67 ± 0.04; P = 0.005, Z = -2.825) at an accuracy level of 67%. The accuracy increased with the number of trials and reached a level of 88% in the last block (trial 41–50). Means of all blocks were significantly different from chance level (trial 11–20: 0.78 ± 0.04, P<0.001, Z = -4.964; trial 21–30: 0.84 ± 0.04, P<0.001, Z = 5.267; trial 31–40: 0.81 ± 0.03, P<0.001, Z = 5.133; trial 41–50: 0.88 ± 0.03, P<0.001, Z = 6.292). Bees of the differential conditioning group chose randomly during the first three blocks (trial 1–10: 0.48 ± 0.05, P = 0.983, Z = -0.131; trial 11–20: 0.56 ± 0.04, P = 0.251, Z = -0.729; trial 21–30: 0.55 ± 0.03, P = 0.268, Z = -0.688) but increased the proportion of correct choices in the course of the training. From the fourth block on, bees significantly preferred the target color over the distractor color (trial 31–40: 0.65 ± 0.05, P = 0.028, Z = -2.109; trial 41–50: 0.67 ± 0.05, P = 0.009, Z = -2.653). Bees of the control group chose randomly among rewarded and unrewarded grey stimuli throughout the entire experiment (trial 1–10: 0.39 ± 0.04, P = 0.078, Z = -1.516; trial 11–20: 0.42 ± 0.03, P = 0.138, Z = -1.170; trial 21–30: 0.45 ± 0.03, P = 0.175, Z = -0.972; trial 31–40: 0.40 ± 0.04, P = 0.083, Z = -1.402; trial 41–50: 0.46 ± 0.04, P = 0.388, Z = -0.792). When testing the bees in the subsequent color choice test for their preference for either blue or turquoise stimuli, bees of the absolute conditioning group (0.52 ± 0.03, P = 0.392, Z = -0.742) and the grey control group (0.48 ± 0.03, P = 0.194, Z = -0.895) chose randomly between stimuli; in contrast, bees of the differential conditioning group chose significantly more often the previously rewarded (correct) stimulus compared to the non-rewarded stimulus (0.67 ± 0.03, P = 0.007, Z = -2.844).

**Fig 3:** Learning performance and color discrimination (choice) test of bees of the three experimental groups. One group of bees was trained with absolute conditioning to one color (against the grey background, black squares). A second group received differential conditioning with one color rewarded and a second color unrewarded (open squares). A third (control) group experienced the training without conditioning to color stimuli (grey squares). See material and methods for the definition of “correct” decision in the grey control group. All groups completed 50 conditioning trials, followed by a choice test, where all bees had to choose between the two colors used in the experiment (blue and turquoise). Horizontal grey dashed line indicates chance level (random choice). All values are mean proportion (±SEM) of correct decisions; **p<0.01; ***p<0.001; ns: not significant; absolute: N = 15; differential: N = 16; grey: N = 12.

### Neuroarchitecture of the MBs

For all experimental groups we found no significant differences in the volume of the calyx or its substructures, the dense collar region and the lip (Fig 4). The mean volume per calyx differed by less than 10% among groups (absolute: 12.7 ± 0.2 x 10^6^ μm^3^; differential: 13.0 ± 0.4 x 10^6^ μm^3^; grey control: 12.5 ± 0.4 x 10^6^ μm^3^; feeder control: 11.9 ± 0.7 x 10^6^ μm^3^) with no statistical significance (P = 0.899, chi^2^ = 0.590). The same was true when considering the volumes of substructures of the calyx; no significant differences were detectable among treatment groups in the lip region (P = 0.872, chi^2^ = 0.705; absolute: 4.6 ± 0.2 x 10^6^ μm^3^; differential: 4.7 ± 0.2 x 10^6^ μm^3^; grey control: 4.7 ± 0.2 x 10^6^ μm^3^; feeder control: 4.4 ± 0.3 x 10^6^ μm^3^) and the dense collar region (P = 0.307, chi^2^ = 3.608; absolute: 4.7 ± 0.1 x 10^6^ μm^3^; differential: 5.1 ± 0.2 x 10^6^ μm^3^; grey control: 4.7 ± 0.2 x 10^6^ μm^3^; feeder control: 4.5 ± 0.3 x 10^6^ μm^3^). For comparison of MG number among groups, data of lALT and mALT regions in the lip were pooled, as no significant differences occurred (MWU; absolute: P = 0.909, Z = -0.115; differential: P = 0.505, Z = -0.666; grey control: P = 0.664, Z = -0.434; feeder control: P = 0.162, Z = -1.398). Between experimental groups, no significant differences were found in the number of MG per 1000 μm^3^ for the lip (P = 0.745, chi^2^ = 1.231; absolute: 36.6 ± 2.3 MG/box; differential: 34.5 ± 1.4 MG/box; grey control: 37.3 ± 2.0 MG/box; feeder control: 36.7 ± 2.3 MG/box) or the dense collar region (P = 0.266, chi^2^ = 3.955; absolute: 62.4 ± 2.8 MG/box; differential: 61.2 ± 2.5 MG/box; grey control: 68.1 ± 2.9 MG/box; feeder control: 63.5 ± 2.9 MG/box; Fig 5A). Estimation of total MG numbers in the lip and dense collar regions also revealed no significant differences among groups, neither for the lip (P = 0.926, chi^2^ = 0.466; absolute: 15.6 ± 0.8 x 10^4^ MG/calyx; differential: 15.9 ± 0.6 x 10^4^ MG/calyx; grey control: 16.6 ± 0.9 x 10^4^ MG/calyx; feeder control: 15.6 ± 1.0 x 10^4^ MG/calyx), nor for the collar (P = 0.310, chi^2^ = 3.587; absolute: 27.3 ± 1.3 x 10^4^ MG/calyx; differential: 31.1 ± 1.5 x 10^4^ MG/calyx; grey control: 30.0 ± 1.0 x 10^4^ MG/calyx; feeder control: 27.6 ± 1.7 x 10^4^ MG/calyx; Fig 5B).

**Fig 4:** Volume of the entire median MB calyx and MB calyx subcompartments (dense collar and lip). No differences were found among experimental groups for the volumes of the entire calyx, dense collar and lip regions. ns: not significant; absolute: N = 13; differential: N = 14; grey: N = 10; feeder: N = 10.

**Fig 5:** Number of microglomeruli per cube (10x10x10μm in size, A) and extrapolated number of MG per calyx (B). No differences in MG numbers were found among groups in any region (dense collar, lip), either when counted per cube or extrapolated to the total number (per calyx). ns: not significant; absolute: N = 13; differential: N = 14; grey: N = 10; feeder: N = 10.

### Possible correlation between behavioral performance and neuroanatomy

Since recent studies have shown a correlation between MG number and olfactory learning and long-term memory in bees and ants [28, 30], we tested for possible correlations between MG density or number, and learning performance, measured as total number of correct landings that was achieved by an individual during the color conditioning phase. We observed evidence for a negative correlation between the number of correct landings in the absolute conditioning group and the MG density in the lip (P = 0.034, r_S_ = -0.588, Fig 6) and the dense collar region (P = 0.044, r_S_ = -0.564). We then extrapolated the mean bouton numbers per box to the volume of the calycal subregions to estimate the total bouton number per calyx lip and collar. Here we observed evidence for correlation between learning performance and MG number in the lip (P = 0.026, r_S_ = -0.613), but not in dense collar region (P = 0.137, r_S_ = -0.435). In contrast, no evidence for a correlation was found for any of the other experimental groups regarding MG density (differential: lip: P = 0.982, r_S_ = —0.007, collar: P = 0.437, r_S_ = -0.226; grey control: lip: P = 0.103, r_S_ = -0.311, collar: P = 0.289, r_S_ = 0.373) and total MG numbers (differential: lip: P = 0.458, r_S_ = -0.216, collar: P = 0.710, r = -0.109; grey control: lip: P = 0.347, r = -0.333, collar: P = 0.184, r = -0.457). However, the observed p-values just failed the significance level α = 0.05 when a Bonferroni correction is applied to account for multiple comparisons (adjusted p<0.025).

**Fig 6:** Correlation between numbers of microglomeruli (MG) and numbers of correct landings in absolute conditioning experiment. Evidence for a correlation between the absolute number of correct landings (from a total of 50 decisions during color conditioning) and an individual’s MG number in both calyx subregions, the lip and the dense collar. Average number of MG per 1000 μm^3^ cube (**A**) and extrapolated to whole volume (**B**). N = 13.

## Discussion

Honeybees are able to associate color stimuli successfully with a sugar reward [9]. However, learning speed and accuracy depend on the type of conditioning [8, 14, 53]. Here we show that bees confronted with an easy absolute conditioning task (one rewarded color stimulus vs. unrewarded background grey) quickly learned the association. No innate preference towards either of the color stimuli was observed, as individuals of the grey control group chose randomly between the respective blue or turquoise stimuli in the final choice test (Fig 3). However, bees trained in the absolute conditioning task failed to discriminate the learned color from a novel, perceptually similar color stimulus (separated by a small color difference of 0.075 hexagon units) when both colors are presented simultaneously in an unrewarded test. When the same two colors were presented to the bees of the differential color conditioning task (one rewarded color vs. one unrewarded color), individuals learned the association much slower, and to a lower level of accuracy; but successfully discriminated between the colors in the subsequent choice test. The difference of discrimination capability of the same set of stimuli in both types of conditioning might be explained by the kind of information that has been learned by the bees during conditioning. Since the amount of information processing by the brain is limited, selective attention enables animals to focus on the most important or easiest accessible features of a given stimulus, rather than learning all potentially available information [56, 57]. Different attention mechanisms might be involved in both types of conditioning, accompanied by a stronger distraction impact of non-target stimuli but higher general attention levels in differential conditioning [8, 14, 58–61], resulting in a slower acquisition curve, but very fine-tuned color discrimination.

At the neuronal level, the MBs were shown to be involved in processing selective attention-like mechanisms in visual discrimination in *Drosophila* [62]. Furthermore, the mushroom bodies have a central function in the formation and long-term storage of associative memories [63, 64]. For olfactory information, memory storage goes along with a modification of the microglomerular organization, i.e. an increase in the connectivity of the neuronal network in the mushroom body lip region ([28] for ants, see [30]). In the present study, we could not find similar effects on the number of microglomeruli in the collar after visual conditioning for respective types of conditioning (Fig 5). It is possible, however, that a potential learning-dependent change in the number of MG after visual conditioning may be masked by the layered structure of the collar (Fig 2C). The MB dense collar region is segmented in five strata [21, 38], which are innervated by neurons from different parts of the inner layers of the medulla [4, 46]. Within the medulla, color information is pre-processed by broad-band, narrow-band and color-opponent neurons [65, 66]. The visual afferent projections from the medulla, which comprises the anterior inferior optic tract (aiot) and the anterior superior optic tracts (asot), innervate the outer rim dense collar [22]. In contrast, lobula projection neurons, particularly the lobula tract, terminate (besides the lip and basal ring) in the loose collar region. All MB input neurons in the collar are color sensitive [22], but whether the different layers are uniformly activated during color learning is currently unknown. However, an accurate estimation of MG in the loose collar is difficult due to its irregularity in structure and MG densities [34]. Compared to the more homogenous conditions in the MB lip, this layered type of projection pattern causes a rather heterogeneous distribution of visually innervated MG in the collar.

A major difference to the olfaction study by [28], in which a learning-induced increase in the number of MG was found in the lip, concerns the conditioning procedure of the bees. While Hourcade *et al*. [28] kept the bees in boxes for seven days after eclosion and maintained them in harnesses for three days in constant darkness after conditioning, we tested free-flying foragers since a non-restrained condition appears essential for fine color learning in bees [67, 68]. Thus, the stimuli-rich natural environment, higher activity rates and motoric requirements, in our case, might have masked a possible effect of the color learning on MG density and number. We aimed to match the natural and ecologically relevant environment in which free flying bees have to find, operate and memorize rewarding flowers. Interestingly, in a recent study on olfactory long-term memory and associated changes in MG organization in the MB lip of leafcutter ants, Falibene *et al*. [30] found a significant increase of MG number two days after learning in freely moving foragers of unknown age. We therefore assume that potentially induced subtle changes of visual MG may remain undetected by our quantification technique due to the complex layered organization of MG in the collar region compared to the more homogenous lip.

The current study found evidence for a negative correlation between number of MG and learning performance (measured as numbers of landings on correct target stimulus) in the absolute discrimination task. This finding suggests that individuals with a lower number of MG perform better in a color learning task. Although the functional significance is currently unclear, one can speculate an effect of experience underlying this correlation: honeybees increase their foraging performance over lifetime (experience; [69]), whereas sensory exposure (synaptic pruning) [43, 70] and increasing age [35] correlate with a decrease in MG density and total number (as also found in two ant species [30, 71]). Therefore, more experienced foragers (with pruned MG density and number) may learn faster than unexperienced individuals (with initially higher MG density and number). The reason why the observed effect was found only in the absolute conditioning group is currently not clear, but might be caused by the fact that the age-dependent increase in foraging performance [69] and hence a higher number of correct landings, is most pronounced and experimentally observed for relatively simple discrimination tasks. Experienced foragers exhibit a higher flower constancy [72], while novices might operate in a more explorative manner (i.e. are more prone to visit novel and unrewarding stimuli). In contrast, performance in more sophisticated tasks, like fine color discrimination learning, might be more sensitive to general differences between learning capabilities of individual bees, which are independent of age or foraging experience but more related to personality [73–75]. However, since the observed correlation was statistically rather weak, we suggest more work on this topic. Additional experiments need to be performed to test the validity and causality by training of age-controlled cohorts in more controlled environments. So far, it remains unresolved whether neuronal correlates of visual information storage for fine color discrimination tasks, rather than the pure processing of that information, are localized in the MBs [22]. The effect of memory formation on the connection between projection neurons from the optic lobes and the dendritic spines from Kenyon cells could potentially be reflected in the ultrastructure of MG (e.g. shape and size of synaptic terminals; [34, 76]). Alternatively, other central brain areas like the lateral protocerebrum (anterior optic tubercle; [23, 77]) and the central complex (*Drosophila*: [78]), or even more peripheral (and upstream) neuropils, like the relatively large medulla [66] and lobula [65], may also play a role in visual memory depending upon the type of conditioning experienced by an individual. The latter may be supported by the observation that first light exposure leads to a significant volume increase in the peripheral optic neuropils in ants [79]. Therefore, the present work underpins that the highly parallel organization of the visual system requires more detailed studies, which aim to link color learning experiments with potentially distributed neuronal plasticity underlying long-term memory formation, to take more brain subdivisions and fine structure (e.g. different collar layers in the calyx) into consideration. Our study provides a potential approach to combine, within subject, complex color learning type behavioral experiments with neuroanatomical analyses to investigate the visual memory trace. In addition, a promising approach to untangle this issue might be color learning under more controlled environmental conditions, using recently developed methods of visual conditioning of the proboscis extension response [68, 80–82] or pharmacological approaches to inhibit protein synthesis prior to MG quantification to prevent neuronal reorganization. Such approaches will be of high value for understanding how these important pollinators make decisions under complex ecological conditions.

## Supporting Information

S1 Table Behavioral data and neuroanatomical measures. (CSV)

## References

[1] ProctorMCF, YeoP. The pollination of flowers. New York: Taplinger Pub; 1972.

[2] BarthFG. Insects and flowers: the biology of a partnership. Princeton: Princeton University Press; 1985.

[3] ReinhardJ, SrinivasanMV, GuezD, ZhangSW. Floral scents induce recall of navigational and visual memories in honeybees. J Exp Bio. 2004; 207(25): 4371–81. 10.1242/jeb.01306 15557023

[4] DyerAG, PaulkAC, ReserDH. Colour processing in complex environments: insights from the visual system of bees. Proc R Soc B. 2011; 278(1707): 952–9. 10.1098/rspb.2010.2412 21147796PMC3049058

[5] Hempel de IbarraN, VorobyevM, MenzelR. Mechanisms, functions and ecology of colour vision in the honeybee. J Comp Physiol A. 2014; 200(6): 411–33. 10.1007/s00359-014-0915-1 24828676PMC4035557

[6] DafniA. Mimicry and deception in pollination. Ann Rev Ecol Syst. 1984; 15: 259–78. 10.1146/annurev.es.15.110184.001355

[7] JersakovaJ, JohnsonSD, KindlmannP. Mechanisms and evolution of deceptive pollination in orchids. Biol Rev Camb Philos. 2006; 81(2): 219–35. 10.1017/S1464793105006986 16677433

[8] Avargues-WeberA, GiurfaM. Cognitive components of color vision in honey bees: how conditioning variables modulate color learning and discrimination. J Comp Physiol A. 2014; 200(6): 449–61. 10.1007/s00359-014-0909-z 24788332

[9] von FrischK. Der Farbensinn und der Formensinn der Biene. SpengelJW, editor. Jena: Verlag von Gustav Fischer; 1914 10.5962/bhl.title.11736

[10] DaumerK. Reizmetrische Untersuchung des Farbensehens der Bienen. Z Vergl Physiol. 1956; 38: 413–78.

[11] von HelversenO. Zur spektralen Unterschiedsempfindlichkeit der Honigbiene. J Comp Physiol. 1972; 80: 439–72. 10.1007/BF00696438

[12] NeumeyerC. Chromatic adaptation in the honeybee: Successive color contrast and color constancy. J Comp Physiol. 1981; 144(4): 543–53. 10.1007/BF01326839

[13] ChittkaL, MenzelR. The evolutionary adaptation of flower colours and the insect pollinators' colour vision. J Comp Physiol A. 1992; 171: 171–81. 10.1007/BF00188925

[14] GiurfaM. Conditioning procedure and color discrimination in the honeybee *Apis mellifera*. Naturwissenschaften. 2004; 91(5): 228–31. 10.1007/s00114-004-0530-z 15146270

[15] DyerA, ArikawaK. A hundred years of color studies in insects: with thanks to Karl von Frisch and the workers he inspired. J Comp Physiol A. 2014; 200(6): 409–10. 10.1007/s00359-014-0913-3 24792861

[16] von FrischK. Tanzsprache und Orientierung der Bienen. Berlin, Heidelberg: Springer-Verlag; 1965 10.1007/978-3-642-94916-6

[17] MenzelR. Untersuchungen zum Erlernen von Spektralfarben durch die Honigbiene (*Apis mellifica*). Z Vergl Physiol. 1967; 56: 22–62. 10.1007/BF00333562

[18] DyerA, GarciaJ. Color Difference and Memory Recall in Free-Flying Honeybees: Forget the Hard Problem. Insects. 2014; 5(3): 629–38. 10.3390/insects5030629 26462830PMC4592575

[19] GiurfaM. The amazing mini-brain: lessons from a honey bee. Bee World. 2003; 84(1): 5–18. 10.1080/0005772X.2003.11099566

[20] DyerAG, ChittkaL. Fine colour discrimination requires differential conditioning in bumblebees. Naturwissenschaften. 2004; 91(5): 224–7. 10.1007/s00114-004-0508-x 15146269

[21] EhmerB, GronenbergW. Segregation of visual input to the mushroom bodies in the honeybee (*Apis mellifera*). J Comp Neurol. 2002; 451(4): 362–73. 10.1002/cne.10355 12210130

[22] PaulkAC, GronenbergW. Higher order visual input to the mushroom bodies in the bee, *Bombus impatiens*. Arthropod Struct Dev. 2008; 37(6): 443–58. 10.1016/j.asd.2008.03.002 18635397PMC2571118

[23] MotaT, GronenbergW, GiurfaM, SandozJC. Chromatic processing in the anterior optic tubercle of the honey bee brain. J Neurosci. 2013; 33(1): 4–16. 10.1523/JNEUROSCI.1412-12.2013 23283317PMC6618620

[24] StrausfeldNJ, HansenL, LiY, GomezRS. Evolution, discovery, and inerpretations of arthropod mushroom bodies. Learn Mem. 1998; 5: 11–37. 10454370PMC311242

[25] MenzelR, GiurfaM. Cognitive architecture of a mini-brain: the honeybee. TRENDS Cogn Sci. 2001; 5(2): 62–71. 10.1016/S1364-6613(00)01601-6 11166636

[26] FahrbachSE. Structure of the mushroom bodies of the insect brain. Annu Rev Entomol. 2006; 51: 209–32. 10.1146/annurev.ento.51.110104.150954 16332210

[27] GiurfaM. Behavioral and neural analysis of associative learning in the honeybee: a taste from the magic well. J Comp Physiol A. 2007; 193(8): 801–24. 10.1007/s00359-007-0235-9 17639413

[28] HourcadeB, MuenzTS, SandozJC, RösslerW, DevaudJM. Long-term memory leads to synaptic reorganization in the mushroom bodies: a memory trace in the insect brain? J Neurosci. 2010; 30(18): 6461–5. 10.1523/JNEUROSCI.0841-10.2010 20445072PMC6632731

[29] GrohC, RösslerW. Comparison of microglomerular structures in the mushroom body calyx of neopteran insects. Arthropod Struct Dev. 2011; 40(4): 358–67. 10.1016/j.asd.2010.12.002 21185946

[30] FalibeneA, RocesF, RösslerW. Long-term avoidance memory formation is associated with a transient increase in mushroom body synaptic complexes in leaf-cutting ants. Front Behav Neurosci. 2015; 9(84). 10.3389/fnbeh.2015.00084 25904854PMC4389540

[31] WitthöftW. Absolute Anzahl und Verteilung der Zellen im Hirn der Honigbiene. Z Morph Tiere. 1967; 61: 160–84.

[32] RösslerW, GrohC. Plasticity of synaptic microcircuits in the mushroom-body calyx of the honey bee In: GaliziaCG, EisenhardtD, GiurfaM, editors. Honeybee neurobiology and behavior. Berlin: Springer Verlag; 2012 p. 141–51.

[33] MaleszkaJ, BarronAB, HelliwellPG, MaleszkaR. Effect of age, behaviour and social environment on honey bee brain plasticity. J Comp Physiol A. 2009; 195(8): 733–40. 10.1007/s00359-009-0449-0 19434412

[34] GrohC, LuZ, MeinertzhagenIA, RösslerW. Age-related plasticity in the synaptic ultrastructure of neurons in the mushroom body calyx of the adult honeybee *Apis mellifera*. J Comp Neurol. 2012; 520(15): 3509–27. 10.1002/cne.23102 22430260

[35] MuenzTS, GrohC, MaisonnasseA, Le ConteY, PlettnerE, RosslerW. Neuronal plasticity in the mushroom body calyx during adult maturation in the honeybee and possible pheromonal influences. Dev Neurobiol. 2015 10.1002/dneu.22290 25784170

[36] MobbsPG. The brain of the honeybee *Apis mellifera*. I. The connections and spatial organization of the mushroom bodies. Philos Trans R Soc Lond B. 1982; 298(1091): 309–54. 10.1098/rstb.1982.0086

[37] AbelR, RybakJ, MenzelR. Structure and response patterns of olfactory interneurons in the honeybee, *Apis mellifera*. J Comp Neurol. 2001; 437: 363–83. 10.1002/cne.1289 11494262

[38] GronenbergW. Subdivisions of hymenopteran mushroom body calyces by their afferent supply. J Comp Neurol. 2001; 436: 474–89. 10.1002/cne.1045 11406827

[39] KirschnerS, KleineidamCJ, ZubeC, RybakJ, GrunewaldB, RösslerW. Dual olfactory pathway in the honeybee, *Apis mellifera*. J Comp Neurol. 2006; 499(6): 933–52. 10.1002/cne.21158 17072827

[40] GrohC, TautzJ, RösslerW. Synaptic organization in the adult honey bee brain is influenced by brood-temperature control during pupal development. P Natl Acad Sci USA. 2004; 101(12): 4268–73. 10.1073/pnas.0400773101 15024125PMC384730

[41] GrohC, AhrensD, RösslerW. Environment- and age-dependent plasticity of synaptic complexes in the mushroom bodies of honeybee queens. Brain Behav Evolut. 2006; 68(1): 1–14. 10.1159/000092309 16557021

[42] GaneshinaO, MenzelR. GABA-immunoreactive neurons in the mushroom bodies of the honeybee: an electron microscopy study. J Comp Neurol. 2001; 437: 335–49. 10.1002/cne.1287 11494260

[43] SchollC, WangY, KrischkeM, MuellerMJ, AmdamGV, RosslerW. Light exposure leads to reorganization of microglomeruli in the mushroom bodies and influences juvenile hormone levels in the honeybee. Dev Neurobiol. 2014; 74(11): 1141–53. 10.1002/dneu.22195 24890265

[44] WüstenbergD, GerberB, MenzelR. Long- but not medium-term retention of olfactory memories in honeybees is impaired by actinomycin D and anisomycin. Europ J Neurosci. 1998; 10: 2742–5.10.1046/j.1460-9568.1998.00319.x9767405

[45] MenzelR. Memory dynamics in the honeybee. J Comp Physiol A. 1999; 185: 323–40. 10.1007/s003590050392

[46] PaulkAC, DacksAM, Phillips-PortilloJ, FellousJM, GronenbergW. Visual processing in the central bee brain. J Neurosci. 2009; 29(32): 9987–99. 10.1523/JNEUROSCI.1325-09.2009 19675233PMC2746979

[47] SpaetheJ, StreinzerM, EckertJ, MayS, DyerAG. Behavioural evidence of colour vision in free flying stingless bees. J Comp Physiol A. 2014; 200(6): 485–96. 10.1007/s00359-014-0886-2 24519371

[48] DyerAG, DorinA, ReinhardtV, GarciaJE, RosaMGP. Bee reverse-learning behavior and intra-colony differences: Simulations based on behavioral experiments reveal benefits of diversity. Ecol Modell. 2014; 277: 119–31. 10.1016/j.ecolmodel.2014.01.009

[49] MorawetzL, SvobodaA, SpaetheJ, DyerAG. Blue colour preference in honeybees distracts visual attention for learning closed shapes. J Comp Physiol A. 2013; 199(10): 817–27. 10.1007/s00359-013-0843-5 23918312

[50] DyerAG, NeumeyerC, ChittkaL. Honeybee (*Apis mellifera*) vision can discriminate between and recognise images of human faces. J Exp Biol. 2005; 208(Pt 24): 4709–14. 10.1242/jeb.01929 16326952

[51] ChittkaL. The colour hexagon: a chromaticity diagram based on photoreceptor excitations as a generalized representation of colour opponency. J Comp Physiol A. 1992; 170: 533–43. 10.1007/BF00199331

[52] DyerAG, ChittkaL. Biological significance of distinguishing between similar colours in spectrally variable illumination: bumblebees (Bombus terrestris) as a case study. J Comp Physiol A. 2004; 190(2): 105–14. 10.1007/s00359-003-0475-2 14652688

[53] DyerAG, NeumeyerC. Simultaneous and successive colour discrimination in the honeybee (*Apis mellifera*). J Comp Physiol A. 2005; 191(6): 547–57. 10.1007/s00359-005-0622-z 15871026

[54] Avargues-WeberA, DeisigN, GiurfaM. Visual cognition in social insects. Ann Rev Entomol. 2011; 56: 423–43. 10.1146/annurev-ento-120709-144855 20868283

[55] ItoK, ShinomiyaK, ItoM, ArmstrongJD, BoyanG, HartensteinV, et al A systematic nomenclature for the insect brain. Neuron. 2014; 81(4): 755–65. 10.1016/j.neuron.2013.12.017 24559671

[56] ZentallTR, RileyDA. Selective attention in animal discrimination learning. J General Psychol. 2000; 127(1): 45–66. 10.1080/0022130000959857010695951

[57] DukasR. Causes and consequences of limited attention. Brain Behav Evolut. 2004; 63(4): 197–210. 10.1159/00007678115084813

[58] ChittkaL, RaineNE. Recognition of flowers by pollinators. Curr Opin Plant Biol. 2006; 9(4): 428–35. 10.1016/j.pbi.2006.05.002 16713328

[59] SpaetheJ, TautzJ, ChittkaL. Do honeybees detect colour targets using serial or parallel visual search? J Exp Biol. 2006; 209(Pt 6): 987–93. 10.1242/jeb.02124 16513924

[60] Avargues-WeberA, de Brito SanchezMG, GiurfaM, DyerA. Aversive Reinforcement Improves Visual Discrimination Learning in Free-Flying Honeybees. PLoS ONE. 2010; 5(10): 1–11. 10.1371/journal.pone.0015370 20976170PMC2955543

[61] MorawetzL, SpaetheJ. Visual attention in a complex search task differs between honeybees and bumblebees. J Exp Biol. 2012; 215(Pt 14): 2515–23. 10.1242/jeb.066399 22723491

[62] van SwinderenB, GreenspanR. Salience modulates 20–30 Hz brain activity in *Drosophila*. Nat Neurosci. 2003; 6: 579–86. 10.1038/nn1054 12717438

[63] HeisenbergM. What do the mushroom bodies do for the insect brain? An introduction. Learn Mem. 1998; 5: 1–10. 10454369PMC311238

[64] MenzelR. Searching for the memory trace in a mini-brain, the honeybee. Learn Mem. 2001; 8(2): 53–62. 10.1101/lm.38801 11274250

[65] PaulkAC, Phillips-PortilloJ, DacksAM, FellousJM, GronenbergW. The processing of color, motion, and stimulus timing are anatomically segregated in the bumblebee brain. J Neurosci. 2008; 28(25): 6319–32. 10.1523/JNEUROSCI.1196-08.2008 18562602PMC3844780

[66] PaulkAC, DacksAM, GronenbergW. Color processing in the medulla of the bumblebee (Apidae: *Bombus impatiens*). J Comp Neurol. 2009; 513(5): 441–56. 10.1002/cne.21993 19226517PMC6783282

[67] NiggebruggeC, LeboulleG, MenzelR, KomischkeB, de IbarraNH. Fast learning but coarse discrimination of colours in restrained honeybees. J Exp Biol. 2009; 212(Pt 9): 1344–50. 10.1242/jeb.021881 19376955

[68] LichtensteinL, SommerlandtFM, SpaetheJ. Dumb and Lazy? A Comparison of Color Learning and Memory Retrieval in Drones and Workers of the Buff-Tailed Bumblebee, *Bombus terrestris*, by Means of PER Conditioning. PLoS ONE. 2015; 10(7): e0134248 10.1371/journal.pone.0134248 26230643PMC4521843

[69] DukasR, VisscherPK. Lifetime learning by foraging honey bees. Anim Behav. 1994; 48: 1007–12. 10.1006/anbe.1994.1333

[70] KrofczikS, KhojastehU, Hempel de IbarraN, MenzelR. Adaptation of microglomerular complexes in the honeybee mushroom body lip to manipulations of behavioral maturation and sensory experience. Dev Neurobiol. 2008; 68(8): 1007–17. 10.1002/dneu.20640 18446779

[71] StiebSM, HellwigA, WehnerR, RosslerW. Visual experience affects both behavioral and neuronal aspects in the individual life history of the desert ant *Cataglyphis fortis*. Dev Neurobiol. 2012; 72(5): 729–42. 10.1002/dneu.20982 21954136

[72] HillPSM, WellsPH, WellsH. Spontaneous flower constancy and learning in honey bees as a function of colour. Anim Behav. 1997; 54: 615–27. 10.1006/anbe.1996.0467 9299046

[73] ScheinerR, BarnertM, ErberJ. Variation in water and sucrose responsiveness during the foraging season affects proboscis extension learning in honey bees. Apidologie. 2003; 34(1): 67–72. 10.1051/apido:2002050

[74] TautzJ, MaierS, GrohC, RösslerW, BrockmannA. Behavioral performance in adult honey bees is influenced by the temperature experienced during their pupal development. P Natl Acad Sci USA. 2003; 100(12): 7343–7. 10.1073/pnas.1232346100 12764227PMC165877

[75] MullerH, ChittkaL. Consistent interindividual differences in discrimination performance by bumblebees in colour, shape and odour learning tasks (Hymenoptera: Apidae: *Bombus terrestris*). Entomol Gen. 2012; 34: 1–8.

[76] KremerMC, ChristiansenF, LeissF, PaehlerM, KnapekS, AndlauerTF, et al Structural long-term changes at mushroom body input synapses. Curr Biol. 2010; 20(21): 1938–44. 10.1016/j.cub.2010.09.060 20951043

[77] MotaT, YamagataN, GiurfaM, GronenbergW, SandozJC. Neural organization and visual processing in the anterior optic tubercle of the honeybee brain. J Neurosci. 2011; 31(32): 11443–56. 10.1523/JNEUROSCI.0995-11.2011 21832175PMC6623125

[78] BarthM, HeisenbergM. Vision affects mushroom bodies and central complex in *Drosophila melanogaster*. Learn Mem. 1997; 4: 219–29. 10.1101/lm.4.2.219 10456065

[79] YilmazA, LindenbergA, AlbertS, GrubelK, SpaetheJ, RosslerW, et al Age-related and light-induced plasticity in opsin gene expression and in primary and secondary visual centers of the nectar-feeding ant Camponotus rufipes. Dev Neurobiol. 2016 10.1002/dneu.22374 .26724470

[80] DobrinSE, FahrbachSE. Visual associative learning in restrained honey bees with intact antennae. PLoS ONE. 2012; 7(6): e37666 10.1371/journal.pone.0037666 22701575PMC3368934

[81] RiverosAJ, GronenbergW. Decision-making and associative color learning in harnessed bumblebees (*Bombus impatiens*). Anim Cogn. 2012; 15(6): 1183–93. 10.1007/s10071-012-0542-6 22837045

[82] JerniganCM, RoubikDW, WcisloWT, RiverosAJ. Color dependent learning in restrained Africanized honey bees. J Exp Biol. 2014; 217(3): 337–43. 10.1242/jeb.091355 24072797

